The article "Personalised Recommendation of PE Network Course Environment Resources Using Data Mining Analysis" was retracted in 2023. Reasons: unreliable results or conclusions; concerns about the data; concerns about the results or conclusions; concerns about the peer review.

# Personalised Recommendation of PE Network Course Environment Resources Using Data Mining Analysis

**DOI:** 10.1155/2022/1032976

**Published:** 2022-08-16

**Authors:** Fanting Min

**Affiliations:** School of Physical Culture, WeiFang University, Weifang 261061, Shandong, China

## Abstract

PE education reform is positively influenced by the creation and use of resources for PE courses as a supplement to and development of traditional teaching strategies. In order to mine the vast amount of data in the network PE curriculum resource system and find useful patterns, this paper uses highly automated DM technology. Additionally, you can forecast users' upcoming actions and suggest particular course resources to them. This recommendation system makes course resources that users might be interested in based on their browsing history, browsing patterns, and browsing preferences. User registration and login, course retrieval, browsing history, course recommendation, and a module for course scoring are among the system's primary features. Studies reveal that this method's recommendation accuracy is up to 96.2 percent, or about 10% higher than that of conventional recommendation methods. The recommendation strategy put forth in this paper has a good recommendation effect, high accuracy, and coverage. It also plays a part in improving the hidden semantic model's accuracy. For individualised curriculum resource recommendations, this recommendation system offers a good solution.

## 1. Introduction

Currently, network teaching is evolving into a cutting-edge educational tool that keeps up with societal and historical changes. The campus network curriculum resource-sharing system is a platform for resource sharing, and we can share resources through the network. Through this system, all users of the campus network can easily and quickly access a variety of curriculum resources [1]. The system generates a massive amount of data, so it's a pressing issue to figure out how to extract useful information from it. This led to the development of recommendation technology, which has since flourished. According to the information that users already possess, recommendation technology makes suggestions for information that the target users might be interested in, making it easier for users to find the information they require [2]. The most popular recommendation algorithms at the moment are the CF (Collaborative Filtering) recommendation algorithm, the content-based recommendation algorithm, the recommendation algorithm based on user-project bipartite graph relationship, and the hybrid recommendation algorithm. Additionally, there are standardised metrics to assess a recommendation system's quality, with accuracy, diversity, novelty, and coverage being the most frequently employed metrics [3]. The problem of “information overload” has become more serious as a result of the growth in resource-sharing platforms, which has led to a steady increase in the number of network-shared resources year after year. Additionally, because online course platforms frequently only offer online teaching videos, the learning effect is minimal [4] and students are unable to interact with teachers offline due to their shifting interests. A PE education reform in colleges and universities should fully utilise the benefits of contemporary distance education, integrate curriculum resources, expand teaching time and space, and enrich teaching methods in order to ensure that PE education can meet the demands of social development in light of the issues with major course teaching in PE, such as the contradiction between venue and training.

The article "Personalised Recommendation of PE Network Course Environment Resources Using Data Mining Analysis" was retracted in 2023. Reasons: unreliable results or conclusions; concerns about the data; concerns about the results or conclusions; concerns about the peer review.

In today's information age, the network has impacted every aspect of our daily lives. In parallel, a significant amount of data has been gathered in all spheres of life thanks to the advancement and widespread use of database and data collection technology. It has become more crucial than ever to figure out how to turn these data into knowledge and information. These requirements are what drive the creation and advancement of DM (Data Mining) technology [5]. Big data mining, storage, and collection are all made possible by DM technology. The value of data can be accurately reflected with the aid of DM tools, which enable people to quickly find hidden patterns in data [6]. Data modelling is a problem that affects DM somewhat independently. DM modelling is a process of gradual improvement after many revisions and requires constant testing in real-world settings. Automatic modelling and model transformation are currently the two main technical topics under discussion in the DM modelling industry [7]. DM technology, which is currently the subject of extensive research and has a wide range of applications in industries such as finance, healthcare, aviation, and transportation, is used extensively in many different fields. The transition from data to knowledge is greatly aided by DM. Based on the analysis of a large amount of data, DM can make inductive arguments and forecast users' behaviour [8]. All network teaching information systems experience “massive data, lack of information” as a common embarrassment after data concentration. Currently, the majority of databases used by the network teaching platform are only capable of low-level operations such as data input, query, and statistics, and they are unable to search through the data for all kinds of useful information [9]. This paper, which is based on DM technology, is concerned with the customised recommendation of PE network course resources from the viewpoint of PE network courses. The following are the main contributions of this paper:

1. In this paper, a specific recommendation process is designed based on the characteristics of curriculum resources. The recommendation system makes course resources that users might be interested in based on their browsing history, browsing patterns, and browsing preferences. Additionally, by using two steps of training, this suggested model addresses the issue of user cold start.
2. In order to address the issue of “user interest drift” in current content-based recommendation algorithms, this paper suggests a method to compute similarity by fusing course similarity and user interest model. The recommendation method in this paper plays a specific role in optimising the accuracy of the hidden semantic model, according to experiments, which also demonstrate the effectiveness, high accuracy, and coverage of the recommendation strategy proposed in this paper.

The article "Personalised Recommendation of PE Network Course Environment Resources Using Data Mining Analysis" was retracted in 2023. Reasons: unreliable results or conclusions; concerns about the data; concerns about the results or conclusions; concerns about the peer review.

## 2. Related Work

At present, the research on recommendation system is quite mature, especially in the field of e-commerce. However, in the field of education, although many researchers pay attention to it and study it, it has not reached the application level as in the field of e-commerce.

Rye S A takes a university's network teaching application system as the background, through the analysis of different types of resource allocation of DM technology based on decision tree algorithm in the construction of school network courses, and introduces the key factors affecting it [10]. Kelly P et al. introduced Web mining technology and its typical application in the campus course resource-sharing system [11]. Lin L used the methods of literature, questionnaires, expert interviews, and logical analysis to investigate and analyse the current situation of information query and utilisation of PE teachers in colleges and universities in the reform of PE curriculum construction [12, 13]. Qi S et al. designed the recommendation process and recommendation algorithm for the specific application environment and the recommendation of course resources in the network teaching platform [14]. To suggest to users products that are appropriate for them, Cothran et al. combined decision tree technology, association rule mining, and Web mining [15]. University PE course resources can be shared in a variety of ways by integrating university PE education resources and developing a shared network platform, according to Meegan S et al. [16]. According to learners' interests and progress, Mei and Li proposed a method to recommend current and future learning materials in real-time. The method is put into practise using three interconnected processes: data collection and processing, learning from nearby students, and learning resource recommendation [17]. Klugman and Beckmann-Mendez combined the basic information of learners and learners' learning styles to improve the CF recommendation algorithm, making the recommendation effect more accurate. At the same time, we have developed and built a recommendation system for small-scale experiments, which provides a reference for the application research of the recommendation system in the field of education [18]. The recommendation system proposed by Shi and Yang applies a hybrid recommendation model based on the neural network [19]. The model includes four modules: content-based recommendation module, item-based CF recommendation module, user-based CF recommendation module, and neural network-based recommendation module. The output of the first three modules is the input of the neural network module, and the neural network module will record the preferences of each user, so as to make personalised recommendations to users.

The article "Personalised Recommendation of PE Network Course Environment Resources Using Data Mining Analysis" was retracted in 2023. Reasons: unreliable results or conclusions; concerns about the data; concerns about the results or conclusions; concerns about the peer review.

Based on the research of related literature and DM technology, this paper focuses on the personalised recommendation of PE network course resources from the perspective of PE network course. This recommended model solves the problem of user cold start by two-step training. Experiments show that the recommendation strategy proposed in this paper has a good recommendation effect, high accuracy, and coverage, and the recommendation method in this paper plays a certain role in optimising the accuracy of the hidden semantic model.

## 3. Methodology

### 3.1. Technical Foundation of DM Personalised Recommendation

Data mining is to mine valuable information from a large amount of data [20]. The data mined by data mining technology is huge and dynamic. A complete DM process mainly includes the following steps: (1) Determine the business object and clearly define the purpose of DM. (2) Data preparation, including data selection, preprocessing and data conversion. (3) Start DM, this step is the core of the whole process. (4) Expression and explanation of results, analysis, and evaluation of results, with the aim of integrating the acquired knowledge into the organisational structure of business information system. Mining association rules are an important method in DM. Mining association rules from potential massive data can obtain data patterns hidden in big data. DM is also a process of knowledge discovery, which includes different steps. In this process, the input is data, and the output is useful information that users expect. Use the data extraction method to sort out scattered network data, get regular knowledge and data, concentrate the data, and transform basic and original data from low level to high level, which provides decision-making basis for student administrators [21]. DM needs some technologies as support, such as massive data collection, powerful multiprocessing computer, and DM algorithm. In the recommendation system based on DM, DM technology is used to analyse user behaviour and user attributes, from which valuable knowledge can be obtained and recommendations can be made. Web access information mining is to mine the access records left by users on the server side when they access the Web. DM architecture is shown in Figure 1.

The article "Personalised Recommendation of PE Network Course Environment Resources Using Data Mining Analysis" was retracted in 2023. Reasons: unreliable results or conclusions; concerns about the data; concerns about the results or conclusions; concerns about the peer review.

How DM results are presented to users is crucial because it is this step that determines how useful the DM results are. The results are typically displayed using a variety of graphical user interfaces and visualisation tools in the final stage of knowledge discovery. The main document classification, automatic generation, clustering, and classification techniques are used in mining. Personalised search engines are possible with the help of these technologies. Ensure that users can access important information with precision and speed. Search engine precision and recall can be increased, search results can be combined, the number of pages can be decreased, and data can be clustered. In terms of the extensive use of information processing technology in PE teaching, college and university PE teachers are still in a relatively archaic state at the moment due to issues such as a lack of information literacy, inability to master and use contemporary information tools, and ignorance of the most recent theories, practises, and trends in PE teaching. In addition, there is a phenomenon known as “importance awareness in place, lack of practical application” that occurs when information acquisition, analysis, processing, transmission, and utilisation are not sufficiently mastered. It is essential to actively encourage collaborative innovation, promote in-depth cooperation among colleges and universities, realise the sharing of PE educational resources among colleges and universities, and realise the customised recommendation of PE network course resources if one hopes to fully realise the functions of PE and maximise the benefits of PE courses in colleges and universities. Users' needs for curriculum resources differ due to differences in their interests. In order to increase user satisfaction, classification technology allows for the provision of personalised services to various users. The campus network curriculum resource-sharing system gains a better understanding of users' interests, forecasts their needs, and makes recommendations for particular curriculum resources to them as a result of the simultaneous mining of potential user data and extraction of user characteristics.

The article "Personalised Recommendation of PE Network Course Environment Resources Using Data Mining Analysis" was retracted in 2023. Reasons: unreliable results or conclusions; concerns about the data; concerns about the results or conclusions; concerns about the peer review.

A personalised recommendation system can offer users a personalised experience. Personalised recommendation services have been implemented by video portals, social networking sites, various shopping sites, and many other websites. Personalised recommendation technology is being studied and employed by many researchers and developers. The recommendation system's basic tenets are as follows: Two users who share similar interests will likely have many of the same items as favourites. Users may enjoy it if the projects are similar to ones they already enjoy and vice versa. The project might appeal to a user if everyone else likes it. The recommendation algorithm is the most important component of the recommendation system, and its approach has a significant impact on how well it functions. The most popular personalised recommendation technology among the various technologies used for recommendations is CF technology. Users can quickly and accurately find resources suitable for their own study among a large number of course resources by using CF technology, which satisfies the users' demand for individualised services. Actually, there is no't a clear line separating CF from other methods in the recommendation system. Some applications of the system's recommendation methods combine the CF algorithm concept. The main goal of CF recommendations based on user data is to identify users who are similar to each other in terms of their item preference data. User-based and project-based CF recommendations are very comparable. In order to determine how similar different resources are to one another and to suggest similar learning resources to users, it also requires historical data. The foundation of CF technology is the interest direction of nearby users, the use of other users' preferences for resource items to determine user similarity, or the prediction of a user's evaluation of a resource based on the shared interests and disinterests of similar users. The system can produce highly accurate personalised recommendations based on these data. It is advised to use CF technology, which offers a high level of personalisation and obvious impact.

### 3.2. Construction of Personalised Recommendation System for PE Course Resources

The goal of the recommendation system is to meet the needs that users have already realised, and at the same time meet the needs that users have not yet realised, or the needs that users have realised but have not shown, so that users can overcome some limitations of themselves. This chapter introduces the design of personalised educational resource recommendation system, including user demand analysis, functional demand analysis, system architecture design, system flow design, database design, and core function design. The acquisition of network data is a process of DM, which requires the information acquirer to have certain retrieval skills and memorising abilities. If the algorithm in the research is directly used in the personalised recommendation module of the curriculum, the performance of the system may be affected because of too much computation. Therefore, in the implementation of the recommendation algorithm, the optimisation of the computational performance of the algorithm should also be considered. This system combines user interests to provide personalised PE course resource recommendations. The majority of its users are system administrators and students. We should fully take into account each learner's unique needs in addition to the needs that are shared by the majority of users when designing this system. On the basis of this, this paper designs and develops a system for recommending PE curriculum resources. The system's storage and persistence layers are found in the database, includes data on database users, learning preferences, resource usage, and users of learning resources who are students. The network resource database was created with the intention of enhancing teaching through the use of its educational resources. Since physical education is different from general education in that it focuses on teaching body movements, students are frequently shown the required movements for PE projects with the aid of videos. Furthermore, the network resource library has a wealth of graphic and audiovisual resources. We can get twice the results with half the teaching effort if we can effectively utilise the PE Network course resources. The process of data selection involves choosing relevant data elements from the original database and other data sources. To choose some column values, users must specifically perform additional analysis and make judgement calls based on understanding the meaning of each data item in the database. The topology diagram of personalised recommendation system for PE course resources is shown in Figure 2.

The article "Personalised Recommendation of PE Network Course Environment Resources Using Data Mining Analysis" was retracted in 2023. Reasons: unreliable results or conclusions; concerns about the data; concerns about the results or conclusions; concerns about the peer review.

The front end of personalised course resource recommendation system includes three modules: user module, course module, and learning materials module. The function of this system can be divided into two parts: The first part is mainly the function of sharing curriculum resources, including the basic function of sharing curriculum resources. The second part is the personalised recommendation function of curriculum resources, mainly including the recommendation function of curriculum resources. The first part provides the basic functional framework for the second part and also generates data for the recommendation of the second part. When designing the course resource recommendation system, this paper mainly analyses the performance requirements from the following aspects: (1) Ease of use requirements. (2) Compatibility requirements. (3) Maintainability requirements. (4) Stability requirements. (5) Scalability requirements. The recommendation system primarily processes data in its work. It is crucial to preprocess the original data for this data processing project. There might be some incorrect or missing data in the initial data for a variety of reasons. The steps of the operation require that the missing data be predicted or supplemented, while the incorrect data can be fixed or eliminated. In order to increase the effectiveness of mining, this paper performs preprocessing, such as transaction identification, data cleaning, session identification, formatting, and deletion of unnecessary information. To offer all students in the school a simple and quick interface of curriculum resources is the goal of the personalised curriculum resource recommendation system. The system's user base is relatively small when compared to that of the enterprise-level course recommendation system. Higher standards for system performance should be set during the system design and development process, though, to enable the system's later expansion. The resource classification entity, which holds all resource classification information, is a description of all the resource classification data on this website. Data cleaning, or the proper handling of incorrect and meaningless data, is what is meant. Error, vacancy, and noise data are three types of problems that can occur with data. Due to the existence of database constraint rules, error data hardly ever appear among them, while vacancy data and noise data are common issues.

The implication form of an association rule is *X*⇒*Y*, and it exists:

(1) $$\begin{array}{c} X\subset I\;Y\subset I\;X\cap Y=\emptyset . \end{array}$$

Confidence, support, and correlation are used as the metrics of association rules, and values between 0% and 100% are used as the interval of confidence and support. The support and confidence of the association rule *X*⇒*Y* are represented by *s* and *α*, respectively. The probability theory expression formulas of support and confidence are as follows:

(2) $$\begin{array}{c} s\left(X\cup Y\right)=P_{r}\left(X\cup Y\right),\\ \alpha \left(X\cup Y\right)=\frac{P_{r}\left(X\cup Y\right)}{P_{r}\left(X\right)}. \end{array}$$

Relevance refers to the degree of correlation between resource *X* and resource *Y*, and its probability theory expression formula is as follows:

(3) $$\begin{array}{c} \sigma_{X,Y}=\frac{\left\{P_{r}\left(X\cup Y\right)\right\}}{\left\{P_{r}\left(X\right)P_{r}\left(Y\right)\right\}}. \end{array}$$

When *P*_*r*_(*X* ∪ *Y*)=*P*_*r*_(*X*)*P*_*r*_(*Y*), *X* and *Y* are independent of each other. The Pearson coefficient is a similarity calculation method based on the correlation coefficient. Generally, in order to make the calculation result accurate, it is necessary to find out the users with common scores. Let the user set *U* be the set of users who commented on both the item *i* and the item *j*, then the corresponding Pearson correlation coefficient calculation formula is:

(4) $$\begin{array}{c} Sim\left(i,j\right)=\frac{\sum_{u\in U}\left(R_{u,i}-{\bar{R}}_{i}\right)\times \left(R_{u,j}-{\bar{R}}_{j}\right)}{\sqrt{\sum_{u\in U}{\left(R_{u,i}-{\bar{R}}_{i}\right)}^{2}\sqrt{\sum_{u\in U}{\left(R_{u,j}-{\bar{R}}_{j}\right)}^{2}}}}. \end{array}$$

Among them, *R*_*u*,*i*_ is the score of the user *u* on the item *i*; ${\bar{R}}_{i}$ is the score of the user *u* set on the item *i*. For a two-dimensional space, according to the vector dot product formula, calculating the cosine similarity between the vector *a* and the vector *b* is to calculate the angle *θ* between the two vectors. Suppose the coordinates of vector *a* and vector *b* are:

(5) $$\begin{array}{c} \left(a_{1},b_{1}\right)\left(a_{2},b_{2}\right). \end{array}$$

Then:

(6) $$\begin{array}{c} \cos\;\theta =\frac{a\cdot b}{\left\|a\right\|\left\|b\right\|}=\frac{a_{1}b_{2}+a_{1}b_{2}}{\sqrt{a_{1}^{2}b_{1}^{2}}\times \sqrt{a_{2}^{2}b_{2}^{2}}}. \end{array}$$

On this basis, extended to a multidimensional space, let *a* and *b* be two *n*-dimensional vectors, where:

(7) $$\begin{array}{c} a\left(a_{1},a_{2},a_{3},\ldots ,a_{n}\right),\\ b\left(b_{1},b_{2},b_{3},\ldots ,b_{n}\right). \end{array}$$

Then the cosine of the angle *θ* between *a* and *b* is equal to:

(8) $$\begin{array}{c} \cos\;\theta =\frac{\sum_{1}^{n}\left(a_{i}\cdot b_{i}\right)}{\sqrt{\sum_{1}^{n}a_{i}^{2}}\times \sqrt{\sum_{1}^{n}b_{i}^{2}}}. \end{array}$$

The similarity of course introduction is calculated by cosine similarity, and the similarity of course attributes is calculated by user interest model. On this basis, the similarity of courses is calculated by weighting, and then the TopN recommendation list is obtained according to the order of numerical value from high to low.

The article "Personalised Recommendation of PE Network Course Environment Resources Using Data Mining Analysis" was retracted in 2023. Reasons: unreliable results or conclusions; concerns about the data; concerns about the results or conclusions; concerns about the peer review.

The user information table, learning style table, and user interest table provide the data for the cosine similarity-based algorithm. The three main steps of the resource recommendation process are: first, data extraction; second, computing the nearest neighbour; and third, resource recommendations. This paper summarises a number of theoretical approaches to data processing based on theoretical research of data preprocessing in the current recommendation system and the test of practise. This method aims to make this theoretical approach universal for data preprocessing in recommendation systems, and it can guide the data processing issues involved in the data preprocessing process of recommendation system, primarily including data selection, supplement, cleaning, and other steps. In this study, the preference weights of various course attributes are dynamically calculated using the user interest model, and the similarity matrix of course attributes is calculated to address the issue of the user's interest drifting over time.

## 4. Result Analysis and Discussion

The system use cases of course personalised recommendation system mainly include resource use cases, message use cases, and search use cases. These use cases show the detailed usage of personalised recommendation system for curriculum resources, including preconditions, ending conditions, input content, and output content. It clearly defines the behaviours triggered by the user's operation under different conditions of wood system, and the conditions for the end of software behaviours. In addition, how to meet the needs of different users is a very important problem that we need to solve urgently, so this paper uses data technology in search engines to build intelligent search engines, thus improving search performance. In order to observe the characteristic values of the output results after mining more carefully, this paper draws the mining results, as shown in Table 1.

This section gathered 8469 pieces of evaluation data from 200 users for 1654 PE curriculum resources. The percentage of user-item scoring matrix items that are not scored is known as the sparse level of the data set, and it is taken into account in the experiment. This experiment has a data sparsity of 0.945. The range of the evaluation value is 1 to 5. The user's preference for the resource increases with value.

In the field of recommendation algorithm, accuracy and recall are the two most basic indicators to measure the recommendation effect, which must be used simultaneously. Accuracy refers to the ratio of recommended related items to the total recommended items. This measure measures the accuracy of the recommendation system. The recall rate refers to the ratio of recommended related items to the total related items, which measures the recall rate of the recommendation system. F-Score comprehensively considers the accuracy and recall. Generally speaking, the higher the value, the more effective the method used. The formula is as follows:

(9) $$\begin{array}{c} \text{F}-\text{Score}=\frac{\left(a^{2}+1\right)\cdot P\cdot R}{a^{2}\cdot \left(P+R\right)}. \end{array}$$

Among them, *P* is the precision rate; *R* is the recall rate; and *a* is the parameter. The F-Scores of different algorithms are compared, and the results are shown in Figure 3.

The article "Personalised Recommendation of PE Network Course Environment Resources Using Data Mining Analysis" was retracted in 2023. Reasons: unreliable results or conclusions; concerns about the data; concerns about the results or conclusions; concerns about the peer review.

The data set is split into a training set and a testing set for the experiment. The algorithm operates on the training set, using the data there to predict the items in the testing set. The following formula represents the MAE (Mean Absolute Error) between the user's actual score and the system's predicted score:

(10) $$\begin{array}{c} \text{MAE}=\frac{1}{c}\sum_{\alpha =1}^{C}|v_{i\alpha }-r_{i\alpha }|. \end{array}$$

Comparing MAE of different algorithms, the results are shown in Figure 4.

Compare the recommendation accuracy of traditional item-based CF and content-based recommendation algorithms with CF algorithm in this paper. The experimental results are shown in Figure 5.

It can be seen from Figure 5 that the CF algorithm in this paper has a large value, which shows that the improved algorithm effectively solves the problem that the traditional similarity algorithm cannot measure the similarity between users and projects when the user-project evaluation matrix is extremely sparse. In the similarity calculation, the effective information is utilised by calculating the union set instead of intersection, and then the score is predicted, and then the similarity is calculated. Based on three different time strategy scoring models, the accuracy calculated by hidden semantic model is shown in Figure 6.

When users visit the homepage of personalised recommendation system for course resources, the recommendation system will calculate a series of resources that users may be interested in and recommend them to users. The recommended resources are calculated according to user preferences, user attributes, and resource attributes. When the user visits the detailed page of course resources, the recommendation system will recommend course resources that are similar to the current resources and may be of interest to the user according to the currently accessed resources and the user's habit records. Collect users' comments on the system recommended in this paper and draw them into a line chart, as shown in Figure 7.

The article "Personalised Recommendation of PE Network Course Environment Resources Using Data Mining Analysis" was retracted in 2023. Reasons: unreliable results or conclusions; concerns about the data; concerns about the results or conclusions; concerns about the peer review.

Freshness means that the products recommended by the recommendation system are not familiar to users and have a certain freshness. Familiarity is the opposite of freshness. Coverage rate describes the ability of the recommendation system to explore the long tail of items, that is, it measures the proportion of items recommended by the recommendation system to the total items. In addition to this proportion, it can generally be measured by calculating the probability of each item being recommended. The freshness, familiarity, and coverage indicators of different recommended systems are shown in Table 2.

The quality of network course construction is one of the important factors that affect the effect of network teaching. The richness and perfection of resource allocation types and quantity of this course can be reflected to some extent by the application of this course. According to experiments in this section, this method's recommendation accuracy can reach up to 96.2 percent, which is roughly 10% higher than that of conventional recommendation methods. This paper describes a method for recommending PE network course resources. As a result, users spend far less time looking for useful information and the system's recommendation effectiveness is increased. This algorithm can predict users' demand for courses and automatically adjust the recommended content.

## 5. Conclusions

Using DM technology to build the recommendation system of network PE curriculum resources can get a lot of useful information, which has practical application value. It can provide great help for the teaching in colleges and universities, and also play a great role in the development of students themselves. PE course resources are bound to promote the further development and improvement of teaching, and improve the network teaching mode; so as to promote school education innovation, deepen teaching reform, promote the application of modern information technology in teaching, share high-quality curriculum resources, and improve the quality of education and teaching. In this paper, DM technology is highly automated to reason and mine the massive information in the network PE curriculum resource system, so as to obtain valuable patterns, predict the future behaviour of users, and recommend specific course resources to them. According to users' browsing records, browsing habits, and preferences, the recommendation system recommends course resources that users may be interested into users. In addition, this recommended model solves the problem of user cold start by two-step training. Experiments show that the recommendation accuracy of this method is up to 96.2%, which is about 10% higher than that of traditional recommendation methods. This algorithm can track users' demand for courses in time and automatically adjust the recommended content, which greatly reduces the time cost for users to find useful information and improves the recommendation efficiency of the system. This recommendation system provides a good solution for personalised recommendation of curriculum resources. However, although this paper has achieved some research results, there are still some shortcomings and areas to be improved in the research process. The accuracy and real-time performance of recommendation system are contradictory. While providing real-time recommendation service, how to effectively improve the quality of recommendation system still needs further research.

The article "Personalised Recommendation of PE Network Course Environment Resources Using Data Mining Analysis" was retracted in 2023. Reasons: unreliable results or conclusions; concerns about the data; concerns about the results or conclusions; concerns about the peer review.

## Figures and Tables

**Figure 1:** DM architecture.

**Figure 2:** Topology diagram of personalised recommendation system for PE network course resources.

**Figure 3:** F-Score comparison of different algorithms.

**Figure 4:** MAE comparison of different algorithms.

**Figure 5:** Comparison of accuracy of different algorithms.

**Figure 6:** Comparison of accuracy of different time strategies.

**Figure 7:** User's subjective evaluation score.

**Table 1:** Detailed list of mining results.

Value	Configuration index ≤360		60< configuration index ≤430		430< configuration index ≤540		540< configuration index	
	Case	Possibility (%)	Case	Possibility (%)	Case	Possibility (%)	Case	Possibility (%)
Animation	1463	5.89	341	4.02	356	8.03	168	7.99
Graphic image	19257	66.58	5604	66.7	2894	71.47	1172	53.64
Sound	476	2.51	115	2.89	198	4.18	0	0
Text	6354	21.97	1359	19.18	176	3.98	598	28.39
Video	3298	3.05	721	7.21	459	12.34	179	9.98
Total node	30848	100	8140	100	4083	100	2117	100

**Table 2:** Index scores of different recommendation systems.

System	Freshness	Familiarity	Coverage rate
CF based on project	3.27	2.87	74.95
Content-based recommendation algorithm	3.71	2.39	81.06
Recommended algorithm in this paper	4.28	1.03	93.27

## Data Availability

The data used to support the findings of this study are available from the author upon request.
